# ω3-PUFAs Exert Anti-Inflammatory Activity in Visceral Adipocytes from Colorectal Cancer Patients

**DOI:** 10.1371/journal.pone.0077432

**Published:** 2013-10-07

**Authors:** Massimo D’Archivio, Beatrice Scazzocchio, Stefania Giammarioli, Maria L. Fiani, Rosaria Varì, Carmela Santangelo, Augusto Veneziani, Annunziata Iacovelli, Claudio Giovannini, Sandra Gessani, Roberta Masella

**Affiliations:** 1 Department Veterinary Public Health and Food Safety, Rome, Italy; 2 Department Hematology, Oncology and Molecular Medicine, Istituto Superiore di Sanità, Rome, Italy; 3 Catholic University “Sacro Cuore”, Rome, Italy; 4 Fabia Mater Hospital, Rome, Italy; Max Delbrueck Center for Molecular Medicine, Germany

## Abstract

**Objective:**

The aim of this study was to correlate specific fatty acid profiles of visceral white adipose tissue (WAT) with inflammatory signatures potentially associated with colorectal cancer (CRC).

**Methods:**

Human adipocytes were isolated from biopsies of visceral WAT from 24 subjects subdivided in four groups: normal-weight (BMI 22.0-24.9 Kg/m^2^) and over-weight/obese (BMI 26.0-40.0 Kg/m^2^), affected or not by CRC. To define whether obesity and/or CRC affect the inflammatory status of WAT, the activation of the pro-inflammatory STAT3 and the anti-inflammatory PPARγ transcription factors as well as the expression of adiponectin were analyzed by immunoblotting in adipocytes isolated from each group of subjects. Furthermore, to evaluate whether differences in inflammatory WAT environment correlate with specific fatty acid profiles, gas-chromatographic analysis was carried out on WAT collected from all subject categories. Finally, the effect of the ω3 docosahexaenoic acid treatment on the balance between pro- and anti-inflammatory factors in adipocytes was also evaluated.

**Results:**

We provide the first evidence for the existence of a pro-inflammatory environment in WAT of CRC patients, as assessed by the up-regulation of STAT3, and the concomitant decrease of PPARγ and adiponectin with respect to healthy subjects. WAT inflammatory status was independent of obesity degree but correlated with a decreased ω3-/ω6-polyunsaturated fatty acid ratio. These observations suggested that qualitative changes, other than quantitative ones, in WAT fatty acid may influence tissue dysfunctions potentially linked to inflammatory conditions. This hypothesis was further supported by the finding that adipocyte treatment with docosahexaenoic acid restored the equilibrium between STAT3 and PPARγ.

**Conclusion:**

Our results suggest that adipocyte dysfunctions occur in CRC patients creating a pro-inflammatory environment that might influence cancer development. Furthermore, the protective potential of docosahexaenoic acid in re-establishing the equilibrium between pro- and anti-inflammatory factors might represent a useful tool for preventive and therapeutic strategies.

## Introduction

The prevalence of obesity has been increasing substantially in the developed countries reaching epidemic proportions [1,2]. This poses a great challenge to global health as obesity represents a main risk factor for a number of chronic degenerative diseases. In addition to cardiovascular diseases and diabetes, epidemiological studies as well as animal models have provided strong evidence that obesity can increase the incidence of many cancers including colorectal cancer (CRC), leukemia, and hepatoma [3-5].

Worldwide, CRC is the third most common cancer accounting for approximately 1.2 million new cases and 608,000 deaths per year [6]. The role of body fatness as a risk factor for CRC has been documented; in particular, it has been recently demonstrated that obesity shows a stronger positive correlation with the risk of developing colon cancer rather than rectal cancer [7-9]. However, the potential mechanisms behind this relation are largely unknown. A critical barrier to progress into the field is represented by the still poor knowledge on how adipose tissue metabolism can impact cancer development.

White adipose tissue (WAT) is increasingly recognized as a complex immunocompetent organ, composed of different cell types among which adipocytes and resident immune cells exhibiting essential secretory and regulatory activities [10]. Obesity disrupts the dynamic role of these cells in energy and immune homeostasis altering the adipokine signaling and leading to a chronic inflammatory status characterized by increased plasmatic levels of inflammatory cytokines such as IL-6 and TNFα [11,12] These factors may synergize to further increase their own concentrations by activating multiple signaling pathways such as STAT3 [13]. This transcription factor, originally identified as a DNA-binding protein, is activated by many cytokines and growth factors and represents a key component in their signaling pathway [14]. Constitutive activation of STAT3 observed in many tumors including colon cancer [15] contributes to oncogenesis by modulating the expressions of a variety of genes involved in proliferation, invasion, metastasis, and angiogenesis [16,17]. In keeping with these observations, a large body of evidence indicates that blocking STAT3 activity suppresses tumor cell growth and induces tumor cell apoptosis [18]. In spite of the key role of STAT3 in oncogenesis, very few studies have explored the activation status of STAT3 in human adipose tissue, providing controversial results [19,20].

To maintain the homeostasis of tissues, STAT3 activity is most likely balanced by other transcriptional regulators with opposite behavior. Among them, peroxisome proliferator-activated receptor γ (PPARγ) is a ligand-activated nuclear hormone receptor with anti-inflammatory role that controls glucose and lipid metabolism. Furthermore, PPARγ is a main regulator of adiponectin expression. Adiponectin, an adipocytokine selectively secreted by WAT, has been shown to inhibit IL-6 secretion and STAT3 activation in colon cancer cells [21] thus attenuating their proliferation [22]. Notably, adiponectin content decreases in obesity [21-23].

Evidence exists that dietary components may influence the inflammatory process and the risk of developing CRC. Fatty acids (FAs) are key components of WAT and their tissue profile closely reflects the dietary intake and/or innate metabolic differences. Changing the nature of the fat consumed may alter the composition of WAT and profoundly influence the FAs available to the body. Interestingly, a potential link between FA composition of WAT and obesity has been highlighted [24]. Given their precursor status to signaling lipid mediators, FAs are major determinants in inflammation. The type of response that FAs induce strongly depends on their biochemical properties, such as number and position of the double bounds. In this regard, different FA families exist, namely saturated FAs, monounsaturated FAs, and ω3 and ω6 polyunsaturated FAs (PUFAs). PUFAs can exert pro- or anti-inflammatory effects depending on their chemical structure. The opposite behaviors of ω3- (anti-inflammatory) and ω6- (pro-inflammatory) PUFAs in modulating several adipose and immune cell functions have been demonstrated [25]. In particular, docosahexaenoic acid (DHA) has been shown to exert a strong anti-inflammatory activity [26].

Aim of this study was to identify alterations of inflammatory status and specific FA profiles of WAT potentially associated with CRC development. The working hypothesis was that WAT represents the initial place where dietary FAs may influence inflammation. FAs could contribute to maintain the proper balance of key transcriptional regulators, thus controlling the inflammatory response of human adipocytes. To define the role of qualitative rather than quantitative changes in WAT FA profiles in tissue inflammation, potentially influencing cancer development, we compared the content of ω3- and ω6-FAs and the inflammatory status of adipocytes isolated from visceral WATs of normal-weight and overweight/obese individuals affected or not by CRC.

We provided evidence for a pro-inflammatory environment in WAT of CRC patients, as assessed by the up-regulation of STAT3, and the concomitant decrease of PPARγ and adiponectin with respect to healthy subjects. This imbalance was independent of obesity degree and correlated with a decreased ω3-/ω6-PUFA ratio. Interestingly, DHA treatment counteracted the altered activation of STAT3 as well as stimulated PPARγ and adiponectin expression.

Taken together our results suggest that adipocyte dysfunctions occur in CRC patients, creating a pro-inflammatory environment that might favor cancer development. Furthermore, the protective potential of DHA in re-establishing the equilibrium between pro- and anti-inflammatory factors might represent a useful tool for preventive and therapeutic strategies.

## Subjects and Methods

### Ethics Statement

The study protocol has been approved by the Ethics Committee of the Istituto Superiore di Sanità. All the subjects gave their informed consent according to the Italian law on this matter (Legislative Decree of the Italian Ministry of Health, January 25, 2001, published in the Official Gazette of April 3, 2001). The participants provided their written informed consent to participate in this study.

### Isolation of human visceral adipocytes

Human visceral adipocytes were collected from anesthetized individuals undergoing abdominal surgery or laparoscopy for CRC or benign conditions. To this purpose 22 subjects affected by CRC were screened to define the eligibility for the study on the basis of the following criteria: histologically proved primary colon adenocarcinoma, stage Duke’s A,B,C/stage I-II-III, any T, any N, M0.

Eighteen subjects undergoing abdominal surgery for gallbladder disease without icterus, umbilical hernia, and uterine fibromatosis were screened to be enrolled as control subjects.

Exclusion’s criteria for all the subjects were: radiotherapy, chemotherapy, steroidal and non steroidal anti-inflammatory therapies, hormonal substitutive or contraceptive therapy, hormonal therapy for any thyroid dysfunctions, drugs or alcohol abuse, diabetes mellitus, chronic renal failure, other neoplastic pathologies, pregnancy, mental disability. Thus, twelve CRC subjects (8 females and 4 males, age 45-67), and 12 control subjects (8 females and 4 males, age 48-72) were enrolled and subdivided in four groups: normal-weight without CRC (NW; n=5); overweight/obese without CRC (Ob; n=7); normal weight with CRC (NWCC; n=5); overweight/obese with CRC (ObCC; n=7). In the NW and NWCC groups, the body mass index (BMI) range was 22.0-24.9 Kg/m^2^. In the Ob and ObCC groups the BMI range was 26.0-40.0 Kg/m^2^, waist circumference >95 cm for men and >80 cm for women. The WAT samplings were performed as previously described [27].

Ten to twenty grams of WAT biopsies were microdissected, rinsed several times in 0.9% NaCl, and digested with 5 ml of Krebs-Ringer solution (0.12M NaCl, 4.7M KCl, 2.5 mM CaCl_2_, 1.2 mM MgSO_4_, 1.2 mM KH_2_PO_4_) containing 20mM HEPES pH 7.4, 3.5% BSA fatty acid-free, 200nM adenosine, 2mM glucose and collagenase (type 1) for 1h (1mg/g adipose tissue) at 37°C in shaking water bath [28]. After collagenase digestion the adipocytes were isolated as previously described [27].

### Treatment of adipocytes with DHA

The adipocytes were treated with 10μM DHA (Sigma Aldrich, St. Louis, MO, USA). DHA was dissolved under nitrogen condition in 100% ethanol to make 10 mM stock solutions, which were stored at -20°C. Stock solutions were diluted in culture media prior to cell treatment. Final concentration of ethanol in treated cells was less than 0.1%. To define the lowest effective concentration of DHA, we carried out preliminary experiments, incubating the isolated adipocytes with different concentration of DHA (1-50µM) for different time periods (6-24h). On the basis of the data obtained (not shown), the experiments were carried out incubating the adipocytes with 10µM DHA for 18h.

### Fatty acids analysis

Total lipids from WAT samples were extracted with chloroform-methanol 2:1 (v/v) according to Folch et al. [29]. FA methyl esters were prepared with 2% methanolic HCl at 100°C for 2h, and extracted with hexane after addition of 2% sodium bicarbonate. All reagents were added with butylated hydroxy toluene (BHT) at the final concentration of 25 mg/L to avoid autoxidation of PUFAs [30].

Fatty acid methyl esters were analyzed using a PerkinElmer Clarus 500 gas chromatograph, equipped with a 60 m x 0.25 mm ID fused-silica capillary column (Rtx 2330, Restek, Bellefonte, PA, USA). Helium was used as carrier gas at 0.8 ml/min. The oven temperature was initially set at 150°C.After 2 min, it was increased to 220°C, at a rate of 3 °C/min, and then to 240°C at 2 °C/min. The column temperature was held at 240°C for 5 min. Injector and detector (FID) were set at 250°C. Peaks were identified by comparison of their retention times with FA methyl ester standards (Supelco 37 Components FAME Mix, Sigma-Aldrich) and quantified by using triheptadecanoin (Sigma-Aldrich) as internal standard (IS).

### Protein determination by Western blot analysis

Whole cell extracts were prepared from adipocytes as previously described [31]. Nuclear protein extracts were prepared by the Nuclear/Cytosol fractionation Kit (Medical & Biological Laboratories, Watertown, LA, USA) according to the manufacturer’s instructions. Immunoblotting analyses were carried out using specific antibodies for STAT3, the tyrosine phosphorylated form of STAT3 (pSTAT3) (Cell Signaling Technology, Danvers, MA, USA), nuclear PPARγ, and adiponectin (Santa Cruz Biotechnology, Santa Cruz, CA, USA). Blots were treated with appropriate secondary antibodies conjugated with horseradish peroxidase (Santa Cruz Biotechnology) followed by ECL detection (Amersham Bio-sciences, Buckinghamshire, UK). Equal loading of proteins was verified by immunoblotting with a goat anti-GAPDH and goat anti-Lamin B antibodies (Santa Cruz Biotechnology) for whole cell and nuclear extracts, respectively. Densitometric analysis was performed using a molecular imager FX (Bio-Rad, Hercules, CA, USA).

### Evaluation of IL-6 secretion

The release of IL-6 was evaluated in the culture media by Elisa kit (R&D Systems Inc, Minneapolis, MN, USA) according to the manufacturer’s instructions.

### Statistical analysis

The results were expressed as means + SEM. Comparisons between 2 groups were carried out by Student’s *t* test. ANOVA followed by Student-Newman-Keuls Multiple Comparison Test were used when >2 groups were compared. Differences were considered significant when P<0.05. Linear regression analysis was performed to determine simple correlation between two variables. P<0.05 was considered as statistically significant.

## Results

### The activation status of STAT3 and PPARγ in adipocytes is differently linked to BMI and cancer condition

The increased risk of CRC linked to obesity might rely on the local aberrant activation of inflammatory pathways establishing a chronic low-grade inflammatory condition, which may predispose to cancer development. To evaluate whether obesity and/or CRC influence the expression/activation of transcription factors critically involved in the regulation of inflammation, the expression of pSTAT3 and of nuclear PPARγ were assessed in visceral adipocytes isolated from the four groups of subjects. As shown in Figure 1, constitutively activated STAT3 was detected in adipocytes independently of subject category. However, higher levels of pSTAT3 were detected in adipocytes derived from CRC subjects with respect to controls. Activated STAT3 was significantly increased in both NWCC and ObCC compared to BMI-matched control subjects (+80% and +151%, respectively; P<0.001). In control subjects (NW and Ob) pSTAT3 levels did not correlate with BMI whereas in CRC patients obesity significantly up-regulated pSTAT3 expression with respect to NWCC (3.47+0.40 OD and 2.15+0.26 OD, respectively; P<0.01) (Figure 1A).

**Figure 1:** Immunoblotting analysis of pSTAT3, PPARγ, and adiponectin. Human visceral adipocytes, collected from the four groups of subjects, were serum-starved for 18 h. Whole cell extracts and nuclear protein extracts were separated by SDS-PAGE and analyzed using anti-pSTAT3 (A), anti-PPARγ (B) and anti-adiponectin (C) antibodies. Results were normalized to STAT3, Lamin B and GAPDH protein content, respectively. NW: normal weight subjects (n=5); Ob: overweight/obese subjects (n=5); NWCC: normal weight with colorectal cancer (n=7); ObCC: overweight/obese with colorectal cancer (n=7). The data are expressed as means ± SEM. *, P<0.05 compared with NW; **, P<0.05 compared with NW and Ob; ***, P<0.05 compared with NW, Ob, and NWCC. Representative blots are shown.

Immunoblotting analysis of nuclear PPARγ, the master regulator of mature adipocyte genes, showed that its expression was significantly affected by both overweight and cancer. In particular, the adipocytes derived from overweight/obese subjects, without or with CRC (1.10+0.15 OD and 1.26+0.19 OD, respectively), as well as those from NWCC subjects (1.73+0.40 OD), showed significantly lower levels of PPARγ compared to NW individuals (3.11+0.23 OD; P<0.01) (Figure 1B). However, in NWCC subjects PPARγ levels were more than 40% higher with respect to all the obese subjects, although the statistical significance was not reached.

In keeping with these results, the expression of adiponectin, a main PPARγ target gene with a well-known anti-inflammatory function, closely reflected the expression of PPARγ being decreased in Ob, NWCC and ObCC individuals with respect to the control NW group. In particular, adiponectin expression was markedly decreased in adipocytes from obese subjects with or without cancer (0.26+0.06 OD and 0.20+0.06 OD, respectively), as compared to NW (1.12+0.31; P<0.01) (Figure 1C).

### The ratio between ω3- and ω6-PUFAs in WAT decreases in CRC subjects irrespective of BMI

To assess whether qualitative changes, other than quantitative ones, in FA stored in visceral WAT potentially associated with CRC occurrence the content of ω3- and ω6- PUFAs was evaluated in visceral WATs isolated from normal-weight and overweight/obese subjects affected or not by CRC.

As shown in Table 1, gas-chromatography analysis did not show any significant difference in the percentage of ω3-PUFAs among the four groups of subjects. Conversely, the percentage of ω6-PUFAs increased in both the obese groups, and reached the statistical significance in ObCC, with respect to both the normal weight groups (P<0.05). Of note, we found a significant decrease in the ω3-/ω6-PUFA ratio not only in the obese groups but also in NWCC with respect to the NW subjects (P<0.05).

**Table 1:** Gas-chromatography analysis of WAT Fatty Acids content in the four groups of subjects.

	**NW**	**Ob**	**NWCC**	**ObCC**
**Saturated FAs (%)**	30+3	32+4	31+3	30+3
**Monounsaturated FAs (%)**	59+4	54+5	58+3	55+6
**ω3-PUFAs (%)**	0.8+0.1	0.7+0.2	0.7+0.2	0.9+0.2
**ω6-PUFAs (%)**	10.6+1.1	12.8+1.4	10.6+0.2	14.0+1.2*^#^
**ω3-/ω6-PUFA ratio**	0.08+0.009	0.056+0.008*	0.065+0.006*	0.059+0.006*

The percentages of saturated and monounsaturated fatty acids (FAs) and ω3- and ω6-polyunsatured fatty acids (PUFAs) were evaluated in visceral adipocytes isolated from normal weight (NW); overweight/obese (Ob); normal weight with colorectal cancer (NWCC), and overweight/obese with colorectal cancer (ObCC) subjects. The data are expressed as means ± SEM. * P<0.05 compared with NW; ^#^ P<0.05 compared with NWCC.

Linear regression analysis aimed at evaluating the relationship existing between obesity degree and ω3-/ω6-PUFA ratio showed an inverse correlation between BMI and ω3-/ω6-PUFA ratio (R=-0.44) (Figure 2A). However, when control and CRC subjects were considered separately, a strong and significant correlation was found in subjects without CRC (R=-0.74; P<0.05) (Figure 2B), but not in those affected by CRC (Figure 2C).

**Figure 2:** Linear regression analysis between ω3-/ω6-PUFA ratio and Body Mass Index (BMI). **A**: all subjects; **B**: subjects without colorectal cancer; **C**: subjects affected by colorectal cancer.

### DHA attenuates STAT3 activation and IL-6 secretion in visceral adipocytes

Since PUFA composition of visceral adipocytes might have a principal role in the imbalance between pro- and anti-inflammatory factors occurring in CRC, we investigated whether exposure of adipocytes to ω3-PUFAs could restore cell homeostasis. To this aim, we assessed the effect of DHA on the expression of pSTAT3, nuclear PPARγ, and adiponectin in adipocytes isolated from the different groups of subjects.

As shown in Figure 3A, DHA significantly (P<0.001) down-regulated pSTAT3 in the adipocytes isolated from Ob (-62%), NWCC (-56%), and ObCC (-59%) subjects with respect to the untreated paired subjects. Conversely, DHA did not exert any effect in adipocytes isolated from the NW group of subjects.

**Figure 3:** Immunoblotting analysis of pSTAT3, and evaluation of IL-6 secretion after DHA treatment. **A**: Human visceral adipocytes, collected from the four groups of subjects, were serum-starved for 18 h. Whole cell extracts were separated by SDS-PAGE and analyzed using anti-pSTAT3 antibody. Results were normalized to STAT3 protein content. The data are expressed as means ± SEM. Representative blots are shown. **B**: IL-6 release was evaluated in the culture media by Elisa as described in Materials and Methods. Data are expressed as means ± SEM. *, P<0.05 with respect to the untreated paired cells. NW: normal weight subjects (n=5); Ob: overweight/obese subjects (n=5); NWCC: normal weight with colorectal cancer (n=7); ObCC: overweight/obese with colorectal cancer (n=7).

Since STAT3 is a key component of signaling pathways leading to the secretion of pro-inflammatory cytokines including IL-6 [32,33], we evaluated whether the DHA-induced modulation of pSTAT3 paralleled a concomitant down-regulation of IL-6. As shown in Figure 3B, the secretion of this cytokine significantly decreased in DHA treated adipocyte cultures in all the groups of individuals (NW, -30%; NWCC, -41%; Ob, -44%; ObCC, -50%) with respect to the untreated paired cells.

### Correlation analyses between ω3-/ω6-PUFA ratio, BMI, and pSTAT3 down-modulation

In order to assess whether a relation exists between ω3-/ω6-PUFA ratio, BMI, and the extent of pSTAT3 decrease after DHA treatment, the correlation coefficients and determinants among these variables were evaluated.

We found a significant inverse correlation between the ω3-/ω6-PUFA ratio and the percentage of pSTAT3 decrease in both control (R=-0.86; P=0.014) and CRC subjects (R=-0.89; P=0.0005) (Figure 4A and B). The finding that DHA treatment was more effective in adipocytes from individuals showing a low ω3-/ω6-PUFA ratio in WAT, suggested that DHA could act by ‘normalizing’ the ω3-/ω6-PUFA ratio to control values.

**Figure 4:** Linear regression analysis between ω3-/ω6-PUFA ratio, Body Mass Index (BMI) and pSTAT3 decrease. Correlation between the ω3-/ω6-PUFA ratio and the percentage of pSTAT3 decrease after DHA treatment in control subjects (n=10) (**A**) and cancer subjects (n=14) (**B**). Correlation between the BMI and the percentage of pSTAT3 decrease after DHA treatment in control subjects (**C**) and cancer subjects (**D**).

As regard the relation between the adiposity degree and the extent of response to DHA treatment, we found a significant positive correlation between BMI and pSTAT3 decrease (R=0.77; P=0.017) in control (Figure 4C) but not in cancer subjects (Figure 4D).

### DHA enhances PPARγ activity and adiponectin expression

To investigate whether the DHA-induced down-regulation of pSTAT3 was accompanied by changes in PPARγ activity and adiponectin content, immunoblotting analysis was performed. As shown in Figure 5, DHA treatment significantly up-regulated both nuclear PPARγ and adiponectin in adipocytes isolated from all the groups of subjects with respect to the paired subjects not receiving the treatment (Figure 5A, B).

**Figure 5:** Immunoblotting analysis of PPARγ, and adiponectin after DHA treatment. Human visceral adipocytes, collected from the four groups of subjects, were serum-starved for 18 h and incubated with 10µM DHA, as described in Material and Methods. Nuclear protein extracts and whole cell extracts were separated by SDS-PAGE and analyzed using anti-PPARγ (**A**) and anti-adiponectin (**B**) antibodies. Results were normalized to Lamin B and GAPDH protein content, respectively. NW: normal weight subjects (n=5); Ob: overweight/obese subjects (n=5); NWCC: normal weight with colorectal cancer (n=7); ObCC: overweight/obese with colorectal cancer (n=7). The data are expressed as means ± SEM. *, P<0.05; **, P<0.01; ***, P<0.01 compared with untreated paired cells. Representative blots are shown.

## Discussion

WAT, namely visceral WAT, is a main source of pro-inflammatory factors, including adipocytokines (e.g. IL-6 and TNFα) and pro-inflammatory chemokines (e.g. CCL2, CXCL8). In obese subjects, WAT is infiltrated by macrophages that participate in the activation of local inflammatory pathways. As a consequence, obesity generates a chronic low-grade inflammation that affects metabolic homeostasis over time. The association of obesity with increased risk, development, and progression of CRC has been established [34]. Epidemiological studies have revealed that overweight and obesity account for 14% of all cancer-related deaths in men and 20% in women [3,35]. For every 2.4 unit increase in BMI, CRC risk increases by 7% [36]. Thus, the rising levels of obesity worldwide are most likely to significantly impact obesity-related CRC in the decades to come. Probably, due to the anatomical proximity of visceral WAT to the intestine in the abdominal cavity, the drainage of its potentially harmful pro-inflammatory products through the portal circulation increases this organ’s vulnerability.

In this study, we provide the first evidence for an ‘inflamed’ visceral WAT in patients affected by CRC.

As regard STAT3 activation, obesity exerted a different influence depending on the presence or not of cancer. In control subjects the increased adiposity was not associated with any increase in pSTAT3 levels. On the contrary, in subjects affected by CRC the presence of increased fat mass seemed to exacerbate the inappropriate activation of STAT3 associated to CRC.

It is well-established that STAT3 plays a crucial role in inducing and maintaining a pro-carcinogenic inflammatory microenvironment, both at the initiation of malignant transformation and during cancer development [37]. STAT3 exerts multiple facet activity by modulating genes relevant for proliferation and survival, as well as those involved in angiogenesis and immunosuppression [38]. STAT3 also regulates the expression of metalloproteinases that enhance migration and metastasis formation [39].

Very few studies have reported the presence of pSTAT3 in human WAT upon adipocyte stimulation with different agents [19,20,40]. Our results add further evidence for the presence of pSTAT3 in WAT, clearly demonstrating that STAT3 is constitutively activated in human adipocytes in the absence of any external stimulation. Notably, while the increase of pSTAT3 was closely related to the presence of cancer rather than obesity, the decrease of activated PPARγ and adiponectin was strongly determined by BMI, in keeping with the low levels of these anti-inflammatory factors even in obese subjects not affected by CRC. In this regard, the marked increase in pSTAT3 levels found in ObCC patients with respect to NWCC subjects might rely on the obesity associated changes in PPARγ and adiponectin levels, establishing a pro-inflammatory environment that promotes STAT3 activation. PPARγ regulates the expression of a variety of genes involved in inflammation, immunity, and metabolism [41], contributing to both metabolic and immune homeostasis. Of note, PPARγ is expressed in many cancers [42-44], and PPARγ agonists have been described to limit growth and induce apoptotic cell death in many human tumors, including CRC [45,46]. However, the exact role of PPARγ in cancer has not been clearly elucidated. A marked reduction in activated PPARγ has been highlighted in the colon of patients with ulcerative colitis, suggesting that PPARγ may contribute to the increased susceptibility to CRC observed in these patients [47]. It has been hypothesized that the anti-cancer effect of PPARγ may rely on its capacity to inhibit pro-inflammatory signals either directly or through the modulation of adipocytokines such as adiponectin [48,49]. An inverse association between adiponectin and cancer, in particular CRC has been suggested. Adiponectin exerts its action directly by inhibiting cancer cell growth [50], or inducing their apoptosis [51], as well as indirectly through pathways related to glucose metabolism, insulin resistance and inflammation [52,53].

Our results provide evidence for the establishment of a pro-inflammatory environment in WAT of CRC subjects, and strengthen the hypothesis that inflamed WAT might influence CRC development. In keeping with our observations, it has been reported that adiponectin, exerting a well-established anti-inflammatory role [54], inhibits IL-6 secretion and STAT3 activation [22], and attenuates proliferation [21] in CRC cells*.*

The significant decrease in the ω3-/ω6-PUFA ratio found in both the obese groups with respect to the NW subjects, together with the finding that the BMI negatively correlated with ω3-/ω6-PUFA ratio, confirmed the link between obesity and a peculiar FA composition of visceral fat most likely predisposing to inflammation [24]. To the best of our knowledge, this is the first demonstration of qualitative changes in FA composition of WAT in CRC subjects independently of BMI, indicating that altered WAT composition linked to an imbalance between pro- and anti-inflammatory factors may take place in cancer patients. Notably, very recently it has been reported that FA distribution of colorectal tissue is significantly different in cancer patients with respect to healthy controls [55].

The critical role of FA composition in driving inflammatory processes in WAT was further supported by the effectiveness of DHA in rebalancing the equilibrium between STAT3 and PPARγ activation in WAT isolated from CRC patients.

Dietary components may influence the inflammatory process and the risk of developing CRC [56,57]. In particular DHA affects several target proteins in chemotherapy resistant SW620 CRC cells in a favorable way [58]; moreover, DHA can block insulin-induced CRC cell proliferation [59].

We found an inverse correlation between ω3-/ω6-PUFA ratio and the extent of pSTAT3 decrease after DHA treatment in both control and cancer subjects, suggesting that DHA was especially effective in subjects with low ω3-/ω6-PUFA ratio. Worth of note, the extent of the response to DHA treatment was independent of BMI in CRC patients. This is consistent with the finding that no correlation existed among BMI and ω3-/ω6-PUFA ratio in CRC patients. Moreover, it should be highlighted that DHA determined a significant decrease in pSTAT3 also in obese control subjects although the basal levels were comparable to the normal weight ones. This effect is most likely due to the pro-inflammatory environment present in obese subjects, at least in part determined by the low levels of PPARγ and adiponectin. Furthermore, obese subjects showed a lower ω3-/ω6-PUFA ratio than NW. By restoring the anti-inflammatory capacities of the cells, DHA might decrease pSTAT3 basal level in adipocytes from obese subjects.

Finally, DHA significantly down-modulated the high levels of IL-6 detected in the adipocytes. This is of utmost importance, because of the close relationship existing between IL-6 secretion and STAT3 activation. In fact, aberrant IL-6 and its down-stream STAT3 signaling in cancer cells has emerged as a major mechanism for cancer initiation and development [60]. However, it is worth of note that DHA induced a significant decrease in IL-6 secretion also in NW subjects, without affecting pSTAT3 levels. This suggests that DHA exerts its anti-inflammatory activity by modulating other pathways involved in IL-6 secretion in addition to the IL-6/STAT3 axis.

In conclusion, our results provide strong evidence that adipocyte dysfunctions of visceral WAT occur in CRC patients, creating a pro-inflammatory environment that might influence cancer development. The onset of this inflammatory condition seems to be influenced by specific alterations of FA profile of WAT. Finally, the protective potential of DHA in re-establishing the equilibrium between pro- and anti-inflammatory factors might represent a useful tool for preventive and therapeutic strategies. However, future research is needed to clarify the mechanism(s) underlying these beneficial effects.
